The article "Human Behavior Recognition in Outdoor Sports Based on the Local Error Model and Convolutional Neural Network" was retracted in 2023. Reasons: signs of a paper mill; compromised peer review; unreliable results or conclusions.

# Human Behavior Recognition in Outdoor Sports Based on the Local Error Model and Convolutional Neural Network

**DOI:** 10.1155/2022/6988525

**Published:** 2022-06-28

**Authors:** Xia Hua, Lei Han, Yang Jiang

**Affiliations:** ^1^Department of Physical Education, China University of Petroleum (East China), Qingdao, Shandong 266580, China; ^2^ZUGO Intelligence Technology (Shen Zhen) Co. Ltd., ZUGO Digital Energy Building Keji First Road High-Tech Zone, Zhuhai, Guandong 519080, China

## Abstract

With the rapid development of the Internet, various electronic products based on computer vision play an increasingly important role in people's daily lives. As one of the important topics of computer vision, human action recognition has become the main research hotspot in this field in recent years. The human motion recognition algorithm based on the convolutional neural network can realize the automatic extraction and learning of human motion features and achieve good classification performance. However, deep convolutional neural networks usually have a large number of layers, a large number of parameters, and a large memory footprint, while embedded wearable devices have limited memory space. Based on the traditional cross-entropy error-based training mode, the parameters of all hidden layers must be kept in memory and cannot be released until the end of forward and reverse error propagation. As a result, the memory used to store the parameters of the hidden layer cannot be released and reused, and the memory utilization efficiency is low, which leads to the backhaul locking problem, limiting the deployment and execution of deep convolutional neural networks on wearable sensor devices. Based on this, this topic designs a local error convolutional neural network model for human motion recognition tasks. Compared with the traditional global error, the local error constructed in this paper can train the convolutional neural network layer by layer, and the parameters of each layer can be trained independently according to the local error and does not depend on the gradient propagation of adjacent upper and lower layers. As a result, the memory used to store all hidden layer parameters can be released in advance without waiting for the end of forward and backward propagation, avoiding the problem of backhaul locking, and improving the memory utilization of convolutional neural networks deployed on embedded wearable devices.

## 1. Introduction

From the advent of computers to the arrival of thousands of households and all walks of life, human beings have increasingly relied on computers for production, life, and entertainment. As humans and computers become more and more inseparable, human-computer interaction has become an indispensable part of human production, life, and entertainment [1–3]. With the development of science and technology, human beings are no longer satisfied with communicating with computers through mechanical keyboards, but they long for a more natural and intelligent way of human-computer interaction. At the same time, the emergence of computer cameras has enabled computers to have the same visual ability as humans, and computer vision has developed rapidly. Humans get inspiration from computer vision, and vision-based human-computer interaction is proposed, which quickly becomes one of the important ways of human-computer interaction, and this gradually affects human production, life, and entertainment [4–6].

The article "Human Behavior Recognition in Outdoor Sports Based on the Local Error Model and Convolutional Neural Network" was retracted in 2023. Reasons: signs of a paper mill; compromised peer review; unreliable results or conclusions.

With the continuous development of the Internet and the accumulation of video data, researchers have proposed many data-driven intelligent processing and analysis techniques. Among them, deep learning technology, as an important technical means in the field of artificial intelligence, is widely used in face recognition, natural language processing, automatic driving, and other fields. Deep learning is a popular direction in machine learning [7]. It models by simulating the physiological mechanism of neurons in the human brain and then processes data in a way similar to human brain learning. With the maturity of computer hardware technology, accelerated by high-performance graphics processors, deep learning has broken the early performance limits in many fields and achieved great gains. Among them, the convolutional neural network in deep learning surpasses the accuracy of manual processing and classification in the recognition and processing tasks of two-dimensional images [8–10]. Convolutional Neural Networks are artificial neural networks based on convolutional operations that excel on image-related tasks. The convolution layer uses the convolution operation to perform operations on the entire image and uses the same weight coefficient for the same feature map, which greatly reduces the amount of parameters of the convolutional neural network, so that the network structure can be kept relatively simple and avoids the complexity of the network model [11–13].

At the same time, the pooling operation of the pooling layer can reduce the number of neurons when constructing the network and maintain the spatial translation invariance of the input data. The convolutional neural network structure has strong scalability, deep layers, and good expressiveness, which provides a foundation for completing the task of visual human-computer interaction. The Convolutional Neural Network (CNN) is a kind of an artificial neural network with convolution operation as the core, which has excellent performance in computer vision-related tasks such as object classification, object detection, semantic segmentation, and image retrieval, and it can satisfy many computer vision tasks [14–16]. Visual needs are widely used in social production and life. In 1994, the convolutional neural network was successfully applied to target detection, but due to problems such as small datasets and hardware technology, the development of target detection based on convolutional neural networks has been stagnant. It was not until 2012, when convolutional neural networks made a major breakthrough in the ImageNet competition, that object detection based on convolutional neural networks began to flourish. Today, convolutional neural networks have surpassed traditional methods and become an important algorithm for target detection. At present, target detection algorithms based on convolutional neural networks can be roughly divided into one-stage target detection algorithms and two-stage target detection algorithms [8, 17].

The article "Human Behavior Recognition in Outdoor Sports Based on the Local Error Model and Convolutional Neural Network" was retracted in 2023. Reasons: signs of a paper mill; compromised peer review; unreliable results or conclusions.

The purpose of this paper is to study the recognition of outdoor human motion data based on wearable sensors, that is, to identify the wearer's motion state through the collected human motion data of wearable sensors. Specifically, first, we design an appropriate wearing position according to the type of action, such as walking, and placing sensors on the wrist and ankle is more comprehensive than the data collected by the waist and neck; secondly, factors such as different ages, genders, and heights need to be considered [18, 19]. We collect abundant human motion data; send the collected motion data into the constructed convolutional neural network for training, learn human motion features, update network parameters, and finally realize motion data recognition. This paper mainly studies the convolutional neural network based on the local error model and applies it to the task of human outdoor motion recognition.

## 2. Method and Theory

### 2.1. Convolutional Neural Network

The Convolutional Neural Network (CNN) is constructed by imitating the biological visual perception mechanism, and it has incomparable advantages in processing images, audio, video, and other data. Compared with the traditional neural network, the difference of the CNN is that it replaces the multiplication operation in the network with the convolution operation. In addition, pooling layers and convolutional layers in the CNN can respond to the translation invariance of input features and identify similar features at different locations.

The basic structure of the CNN is mainly composed of convolutional layers, pooling layers, and fully connected layers. Among them, the neuron is the basic unit of the convolutional layer. During network training and network learning, neurons acquire their corresponding weight values. The neurons between different convolutional layers implement data mapping through nonlinear functions and then aggregate the data through the pooling layer and pass the simplified feature data to the next layer. Finally, the fully connected layer maps the feature information to the sample label space and makes a behavior recognition decision on it.

The article "Human Behavior Recognition in Outdoor Sports Based on the Local Error Model and Convolutional Neural Network" was retracted in 2023. Reasons: signs of a paper mill; compromised peer review; unreliable results or conclusions.

The convolution layer performs the convolution operation on the data information to obtain the semantic features existing in the data, and its function in the image sequence is to extract the underlying features in the image. Convolutional layers of different depths have different input data. Among them, the input data of the top convolution layer are a sequence of video images, and the middle layer uses the feature data of the previous layer as the input. It is worth noting that each convolution kernel corresponds to a feature result. All convolution kernels have their own weight coefficients and offsets, and these parameters are shared during network training or prediction. The convolution of the first layer takes a sequence of video frames or images as input. When performing a convolution operation, the layer data are scanned according to the stride of the convolution kernel, and it is convolved with the convolution kernel. The convolution of the first layer can obtain low-level features in the image, such as contour lines, and then process the convolution results through a nonlinear function and then output feature data. The feature data of this layer constitute the features of the first layer. The convolutional layer in the middle layer uses the output of the upper layer as the input of this layer.

The weight parameters and the carried bias in the convolution kernel will be continuously trained and updated iteratively according to the input data. In order to reduce the number of updates of the training parameters and accelerate network training, different perceptual fields can be used to perform convolution operations on the feature maps. The convolution of the middle layer is to reprocess the feature information of the upper layer to obtain more advanced semantic features. The essence of pooling is to compress the convolutional feature map. The operation is to select a part of the convolutional feature map of a certain size, discard the redundant feature data according to the correlation of the features, and select the most representative data as new feature data. The pooling operation can reduce and compress the huge feature data and change the output data volume of the network layer. Generally speaking, the pooling layer is next to the convolutional layer, and the input data of the pooling layer are the convolutional feature data of the previous layer. The pooling operation realizes the reduction of the dimension of the convolutional feature data, while reducing the interference caused by data changes or noise. After convolutional layer convolution processing and pooling layer filtering and aggregation, the input data become a local feature map, and when the network finally outputs, it needs to splice these local features to achieve final feature fusion, and the fully connected layer completes this step. In the final decision of the network, the fully connected layer expands the feature map obtained after final pooling in turn and builds it into a connection vector as the network input of this layer. At this time, the feature map is transformed from a three-dimensional structure to two-dimensional data; that is, the last input of the network is a two-dimensional vector, which is passed to the next layer after being processed by the excitation function. The fully connected layer comprehensively considers all features. The calculation process of the convolution layer and the pooling layer is the same, and the calculation operations are shown in formulas (1) and (2).

(1) $$\begin{array}{c} {\text{High}}_{\text{out}}=\frac{{\text{High}}_{\text{in}}+2\times {\text{High}}_{\text{padding}}-{\text{High}}_{\text{kernet}}}{{\text{High}}_{\text{stride}}}+1, \end{array}$$

(2) $$\begin{array}{c} {\text{Wide}}_{\text{out}}=\frac{{\text{Wide}}_{\text{in}}+2\times {\text{Wide}}_{\text{padding}}-{\text{Wide}}_{\text{kernet}}}{{\text{Wide}}_{\text{stride}}}+1. \end{array}$$

Among them, High_in_ and Wide_in_ are the height and width of the input feature map or input image data, Wide_out_ is the height and width of the output map feature map, and High_padding_, Wide_padding_ are the input data. The height and width of the padding, High_kernet_, Wide_kernet_ are the height and width of the convolution kernel, and  High_stride_, Wide_stride_ are the height and width of the convolution kernel moving step.

The article "Human Behavior Recognition in Outdoor Sports Based on the Local Error Model and Convolutional Neural Network" was retracted in 2023. Reasons: signs of a paper mill; compromised peer review; unreliable results or conclusions.

In the field of video behavior recognition, the most direct processing method is to cut out a specific video frame from the video data and perform behavior recognition according to the data of the video frame. Compared with the direct recognition task of video data, this method of intercepting video frames and reprocessing greatly reduces the amount of computation. When the network is trained and learned, the intercepted video frames are directly sent to the network to extract features, and then the behavior category in the video is judged. There are very obvious defects in this method; that is, the interception of video frames greatly affects the determination of behavior categories. If the intercepted video frames do not have the representativeness of behavior, it will lead to misjudgment to a large extent, and the single action of some actions will lead to misjudgment. The frame images are very similar, which will lead to extremely poor recognition. Therefore, how to let the neural network learn the continuous motion information in the video image sequence is very important, and effective feature extraction can effectively complete the action recognition.

### 2.2. Algorithm Research on Layer-by-Layer Error Training

At present, the wearable sensor human motion recognition system based on the convolutional neural network usually uses the global error function for back-propagation to achieve the purpose of network parameter update. In the above process, all hidden layer parameters in the neural network need to be stored in the memory and cannot be released before forward propagation and back propagation are completed, which is called the return lock phenomenon. Global neural network training needs to store global reverse gradient flow parameters, which greatly occupies computer resources, resulting in slow convergence and long training time. The backhaul locking phenomenon hinders the reuse of memory, which seriously restricts the application of wearable devices with limited resources in the field of human motion recognition. In addition, training methods based on global errors are widely questioned by biologists due to their biological inexplicability.

In this paper, the idea of a local error model is proposed in the field of outdoor motion recognition based on wearable sensors. The traditional global error is replaced by the local training error to avoid storing the global reverse gradient flow parameters. The layer-by-layer training error is used to realize the layer-by-layer parameter update and finally complete the convolutional neural network human motion recognition system with high memory utilization, fast training speed, and large accuracy improvement. By designing the local error model, we apply it to all hidden layers and realize the parameter update in small batches through the layer-by-layer training mode. The problem that the global error cannot update the network parameters in small batches is solved, thereby accelerating the convergence speed of the entire network model. The construction of the layer-by-layer local error function mainly includes two error functions, the similarity matching function and the cross-entropy function (Figure 1).

The article "Human Behavior Recognition in Outdoor Sports Based on the Local Error Model and Convolutional Neural Network" was retracted in 2023. Reasons: signs of a paper mill; compromised peer review; unreliable results or conclusions.

The fully connected layer outputs *Y* as the comparison label of *S*(*h*), and its mean square error is

(3) $$\begin{array}{c} L_{\text{mse}}=S\left(h\right)-S{\left(Y\right)}_{F}^{2}. \end{array}$$

At the same time, the real label *Y* is used as the fully connected layer to output the $\dot{Y}$ label, and its cross entropy loss function is calculated

(4) $$\begin{array}{c} L_{c}=\text{CrossEntropy}\left(Y,\dot{Y}\right). \end{array}$$

According to the weight ratio, the local training error is finally obtained

(5) $$\begin{array}{c} L=\alpha L_{\text{mse}}+\left(1-\beta \right)L_{c}, \end{array}$$

where *α* and *β* are constants.

This paper uses the local error signal to complete the update of the current network parameters. The global error gradient is replaced by a single layer-by-layer error signal. The gradient flow parameters stored in the computer memory are only the gradient flow parameters of the network in this layer, which greatly reduces the amount of computer resources and speeds up the training speed of the neural network.

## 3. Results and Discussion

Hyperparameters stored in the model include training batches, optimizers, and learning rates. This paper mainly explores the influence of the local error algorithm on the model, so the hyperparameter adjustment in the experiment is not the main research focus. In addition, the setting of the joint weight parameter in the model affects the recognition performance of the local error method, so the joint weight parameter needs to be adjusted for multiple verifications. The joint weight parameter experiment selects the public human motion data set UCI-HAR and determines its best performance point by adjusting different joint weight parameter values a, as shown in Figure 2. The abscissa represents different joint weight parameters a, and the ordinate represents the size of the error. The ordinate of the experiment is the average error of 50 batches after convergence. It can be seen from the experiments that the effect of the joint weight parameter on the model performance is nonmonotonic, and the optimal recognition result can be obtained when the joint weight parameter is set to 0.99. Therefore, all experiments in this topic uniformly set the joint weight parameter to 0.99.

### 3.1. Performance Metrics and Evaluation Criteria

Common indicators to measure the generalization ability of models include the error rate, precision, precision rate, and recall rate. Human motion classification is more concerned with the proportion of correctly classified samples to the total samples, that is, the accuracy. The formula expression is

(6) $$\begin{array}{c} P=\frac{\text{TP}}{\text{TP}+\text{FP}}, \end{array}$$

where TP and FP represent true positives and false positives, respectively. In a natural environment, it is difficult to repeatedly collect specific human movements, which will lead to an unbalanced distribution of motion data types. It is unscientific to use accuracy as a single performance indicator for judging the generalization ability of a model.

The article "Human Behavior Recognition in Outdoor Sports Based on the Local Error Model and Convolutional Neural Network" was retracted in 2023. Reasons: signs of a paper mill; compromised peer review; unreliable results or conclusions.

### 3.2. Experiment and Performance Analysis

In order to evaluate the performance of the convolutional neural network algorithm based on the local error, this experiment uses public datasets including UCI-HAR dataset, OPPORTUNITY dataset, UniMib-SHAR dataset, and PAMAP2 dataset. We use a convolutional neural network with a global error with the same parameter settings as a benchmark and compare a single cross-entropy error model Pred, a single similarity matching error model Sim, and our local error training model PredSim. The specific experimental results are as follows:

#### 3.2.1. UCI HAR Dataset Experiment

Table 1 is the model parameter setting table of UCI HAR, which includes parameter settings such as the number of convolution kernels, training period, training batch, and learning rate.

In experiments, the proposed local error identification model is compared with three baseline models, as shown in Figure 3. In Figure 3, the abscissa Epoch is the training period, and the ordinate Error is the loss error. Experiments show that the recognition effect of a single cross-entropy error model is not as good as that of the global error convolutional neural network model, and the single similarity matching model is approximately close to the global error model. In particular, the proposed local error model outperforms the three baseline models over the entire training epoch and remains stable. On the other hand, on the basis of the same learning rate setting, the proposed local error model converges faster than the other three baseline models.

#### 3.2.2. Experiment on the OPPORTUNITY Dataset

Table 2 is the model parameter setting table of OPPORTUNITY, which includes parameter settings such as the number of convolution kernels, training period, training batch, and learning rate.

In the experiment, the NULL category of the OPPORTUNITY dataset accounts for 72.28% of the dataset. Unbalanced datasets that are too high for a single category will affect the recognition effect of small categories, and their recognition accuracy will be higher than that of the corresponding balanced datasets. As shown in Figure 4, our local error model has faster convergence speed and more stable recognition accuracy than the three baseline methods. On the other hand, the recognition accuracy of the benchmark model based on the global error signal is much lower than that based on the local error signal in the testing process.

The article "Human Behavior Recognition in Outdoor Sports Based on the Local Error Model and Convolutional Neural Network" was retracted in 2023. Reasons: signs of a paper mill; compromised peer review; unreliable results or conclusions.

#### 3.2.3. UniMib-SHAR Dataset Experiment

Table 3 is the model parameter setting table of UniMib-SHAR, which introduces the parameter settings such as the number of convolution kernels, training period, training batch, and learning rate. The learning rate is a dynamic learning rate strategy, using learning rates of 0.003, 0.0015, and 0.0009 at 7.5%, 5%, and 87.5% of the training period, respectively.

In experiments, the proposed local error identification model is compared with three baseline methods, as shown in Figure 5. Experiments show that the single similarity matching error model can still achieve significant improvement over the standard convolutional neural network model baseline, and the convergence speed is much faster than the standard convolutional neural network model. When combined with local error signals, the test error can still maintain a high level. When the training period reaches 150, the Sim model and the Predsim model basically converge, and the training error curve will warp back.

#### 3.2.4. PAMAP2 Dataset Experiment

Table 4 is the model parameter setting table of PAMAP2, and Table 4 details the parameter settings such as the number of convolution kernels, training period, training batch, and learning rate.

In experiments, the proposed local error identification model is compared with three baseline methods, as shown in Figure 6. Experiments show that the proposed local error method can consistently surpass the other three baseline methods in recognition accuracy in 500 training cycles, and the convergence speed is much faster than the standard convolutional neural network model, as shown in Figure 6. Compared with other experimental error curves, the four test error curves in the training process of this experiment have a large jitter in the early stage. In fact, the PAMAP2 dataset has many types of human motions, including several types of human motions that are difficult to collect, such as cleaning with vacuum cleaners and ironing clothes. The problem of class imbalance leads to the majority class in the initial stage of neural network training, and the update of parameters and weights revolve around the majority of motion classes. The recognition accuracy of a few human motion types fluctuates irregularly, and it is difficult to achieve a balance between the comprehensive recognition accuracy and a small number of motion types. Therefore, the test error curve in the pretraining stage has a large random jitter.

The article "Human Behavior Recognition in Outdoor Sports Based on the Local Error Model and Convolutional Neural Network" was retracted in 2023. Reasons: signs of a paper mill; compromised peer review; unreliable results or conclusions.

## 4. Conclusion

1. This paper first introduces the principle of the convolutional neural network and introduces the neural network structure such as convolutional layer and pooling layer in detail. Then, the process and principle of the local error algorithm are introduced, and the local error convolutional neural network model is designed and built.
2. This paper conducts a comparative analysis of the performance of four public datasets and baseline models. The problems such as jitter and back warping of the test error curve appearing in the experiment are discussed. The final local error algorithm achieves high recognition performance in four public human motion datasets with high memory utilization.

## Figures and Tables

**Figure 1:** Partially trained model.

**Figure 2:** The effect of joint weight parameters.

**Figure 3:** Error comparison between the UCI HAR local error model and the baseline model.

**Figure 4:** Error comparison between the OPPORTUNITY local error model and the baseline model.

**Figure 5:** Comparison of errors between the UniMib-SHAR local error model and the baseline model.

**Figure 6:** The error comparison of the PAMAP2 local error model and the baseline model.

**Table 1:** UCI HAR model parameter settings.

Model parameters	Parameter setting

Number of sliding convolution layers	3
Number of convolution kernels	128, 256, 384
Training period	500
Training batch	200
Dynamic learning rate	(4,1,0.9,0.7,0.5) × 10^−3^

**Table 2:** OPPORTUNITY model parameter settings.

Model parameters	Parameter setting

Number of sliding convolution layers	3
Number of convolution kernels	128, 256, 384
Training period	500
Training batch	200
Learning rate	0.001

**Table 3:** UniMib-SHAR model parameter settings.

Model parameters	Parameter setting

Number of sliding convolution layers	3
Number of convolution kernels	128, 256, 384
Training period	500
Training batch	200
Learning rate	(3,1.5,0.9) × 10^−3^

**Table 4:** PAMAP2 model parameter settings.

Model parameters	Parameter setting

Number of sliding convolution layers	3
Number of convolution kernels	128, 256, 384
Training period	500
Training batch	200
Learning rate	0.0005

## Data Availability

The figures and tables used to support the findings of this study are included within the article.
